This article has been retracted.

# The Risk Model Based on the Three Oxidative Stress-Related Genes Evaluates the Prognosis of LAC Patients

**DOI:** 10.1155/2022/4022896

**Published:** 2022-06-23

**Authors:** Qiang Guo, Xiao-Li Liu, Hua-Song Liu, Xiang-Yu Luo, Ye Yuan, Yan-Mei Ji, Tao Liu, Jia-Long Guo, Jun Zhang

**Affiliations:** ^1^Department of Cardiothoracic Surgery, Taihe Hospital, Hubei University of Medicine, Shiyan 442012, Hubei Province, China; ^2^Department of Ultrasound, The People's Hospital of Jianyang City, Jianyang 641400, Sichuan Province, China

## Abstract

**Background:**

Oxidative stress plays a role in carcinogenesis. This study explores the roles of oxidative stress-related genes (OSRGs) in lung adenocarcinoma (LAC). Besides, we construct a risk score model of OSRGs that evaluates the prognosis of LAC patients.

**Methods:**

OSRGs were downloaded from the Gene Set Enrichment Analysis (GSEA) website. The expression levels of OSRGs were confirmed in LAC tissues of the TCGA database. GO and KEGG analyses were used to evaluate the roles and mechanisms of oxidative stress-related differentially expressed genes (DEGs). Survival, ROC, Cox analysis, and AIC method were used to screen the prognostic DEGs in LAC patients. Subsequently, we constructed a risk score model of OSRGs and a nomogram. Further, this work investigated the values of the risk score model in LAC progression and the relationship between the risk score model and immune infiltration.

**Results:**

We discovered 163 oxidative stress-related DEGs in LAC, involving cellular response to oxidative stress and reactive oxygen species. Besides, the areas under the curve of *CCNA2*, *CDC25C*, *ERO1A*, *CDK1*, *PLK1*, *ITGB4*, and *GJB2* were 0.970, 0.984, 0.984, 0.945, 0.984, 0.771, and 0.959, respectively. This indicates that these OSRGs have diagnosis values of LAC and are significantly related to the overall survival of LAC patients. *ERO1A*, *CDC25C*, and *ITGB4* overexpressions were independent risk factors for the poor prognosis of LAC patients and were associated with risk scores in the risk model. High-risk score levels affected the poor prognosis of LAC patients. Notably, a high-risk score may be implicated in LAC progression via cell cycle, DNA replication, mismatch repair, and other mechanisms. Further, *ERO1A*, *CDC25C*, and *ITGB4* expression levels were related to the immune infiltrating cells of LAC, including mast cells, NK cells, and CD8 T cells.

**Conclusion:**

In summary, *ERO1A*, *CDC25C*, and *ITGB4* of OSRGs are associated with poor prognosis of LAC patients. We confirmed that the risk model based on the *ERO1A*, *CDC25C*, and *ITGB4* is expected to assess the prognosis of LAC patients.

## 1. Introduction

Oxidative stress is a state of imbalance between the oxidation and antioxidant effects in the human body. Increasing the neutrophil infiltration and oxidative intermediates by oxidative stress contributes to disease occurrence. Current studies indicate that oxidative stress regulates cancer progression [1–3]. For instance, interleukin-8 (IL-8) is a bridge between inflammation and oxidative stress-induced death of cancer cells. IL-8 overexpression promotes the proliferation of prostate cancer cells and inhibits cell apoptosis. IL-8 and mTOR reduce cellular oxidative stress by suppressing GSK-3*β* expression and protecting prostate cancer cells [3]. Excessive reactive oxygen species (ROS) production triggers oxidative stress, potentially causing cancer. Overexpression of *miR-526b/miR-655* promotes the invasive capacity of breast cancer (BC) cells. *miR-526b* and *miR-655* regulate the *TXNRD1* expression to cause oxidative stress in BC [4].

Oxidative stress plays a significant role in cancer progression [5–8]. Twist-related protein 2 (*TWIST2*) modulates tumorigenesis, tumor progression, and epithelial-mesenchymal transformation (EMT). *TWIST2* is substantially downregulated in lung cancer tissues and cells. *TWIST2* overexpression causes apoptosis, promotes the expression of E-cadherin protein, and inhibits the expression of N-cadherin, vimentin, and slug proteins. Besides, *TWIST2* causes oxidative stress in lung cancer cells and inhibits lung cancer progression by modulating the *FGF21*-mediated *AMPK/mTOR* signaling pathway [5]. The nuclear factor, erythroid-derived 2 (*Nrf2*), is a hub transcription factor for cell adaptation and defense against oxidative stress. Oxidative stress reduces *Nrf2* SUMOylation and promotes LAK cell invasion and migration. SUMOylation of *Nrf2* increases its antioxidant capacity and reduces the level of ROS in LAC cells. Decreased SUMOylation of *Nrf2* and increased ROS stimulate the JNK/c-Jun signaling axis to enhance cell migration and cell adhesion, as well as promote LAC cell invasion [7]. At present, risk score models are utilized to evaluate the prognosis of cancer patients [9–11]. Herein, the oxidative stress-related genes (OSRGs) were downloaded from the official website of Gene Set Enrichment Analysis (GSEA). The expression levels of OSRGs were identified in LAC tissues of The Cancer Genome Atlas (TCGA) database. Thereafter, we investigated oxidative stress-related differentially expressed gene (DEG) mechanisms. The contributing DEGs to poor prognosis in patients with LAC were screened using the Kaplan-Meier (K-M) survival analysis, receiver operating characteristic (ROC) analysis, and Cox analysis AIC method. Subsequently, we constructed the risk score model and nomogram of LAC patients and then identified the roles of the risk score model in the progression and prognosis of LAC patients.

## 2. Materials and Methods

### 2.1. Acquisition of OSRGs

The OSRGs were searched on the online GSEA website (http://www.gsea-msigdb.org/gsea/index.jsp) [12]. The input keywords included oxidative stress and the 32 gene sets related to oxidative stress. All 32 gene sets were extracted, and the remaining genes, after eliminating the duplicate genes, were defined as OSRGs.

### 2.2. Oxidative Stress-Related the DEGs in LAC

The gene expression data of 594 LAC patients with FPKM type were downloaded from the official website of TCGA (https://portal.gdc.cancer.gov/) database. Of these, 59 were normal lung samples, whereas 535 were LAC samples. The expression data of OSRGs in 594 samples were retrieved. The expression of OSRGs in LAC tissues was identified by the limma package. The inclusion criteria were |logFC| = 1 and false discovery rate (FDR) < 0.05, which were defined as the oxidative stress-related DEGs.

### 2.3. Biological Functions in the Oxidative Stress-Related DEGs

Gene Ontology (GO) annotation and Kyoto Encyclopedia of Genes and Genomes (KEGG) signaling pathway analysis were used to analyze the roles and mechanisms of multiple genes [13, 14]. The biological process (BP), cell composition (CC), and molecular function (MF) of the oxidative stress-related DEGs were explored through GO annotation. The screening standard was adjusted to *P* < 0.05. The signaling mechanisms involved in the oxidative stress-related DEGs were analyzed using the KEGG signaling pathway, and the screening standard was adjusted to *P* < 0.05.

### 2.4. Protein-Protein Interaction (PPI) Network between the Oxidative Stress-Related DEGs

The online STRING (version: 11.5) website (https://string-db.org/) was used to observe the interaction between multiple genes [14]. Therefore, the oxidative stress-related DEGs were entered into the STRING database to display the PPI network between the oxidative stress-related DEGs. The screening criteria of the PPI network is the combined score > 0.4. The visualization of the PPI network of the oxidative stress-related DEGs was further enhanced by the Cytoscape (version: 3.8.2) software. The oxidative stress-related DEGs were enriched and analyzed using the MCODE method.

### 2.5. The Prognostic Values of the Oxidative Stress-Related DEGs

The prognostic data and clinicopathological features of 522 patients with LAC were downloaded from the official website of the TCGA database. After excluding 522 patients with incomplete prognostic information of LAC, the oxidative stress-related DEGs of 535 patients with LAC were matched with the prognostic information of LAC patients. By grouping the median values of the oxidative stress-related DEGs, the roles of the DEGs in the overall survival (OS) of patients with LAC were investigated by K-M survival analysis. The screening standard was set at *P* < 0.001.

### 2.6. Construction of the Prognostic Nomogram of the Oxidative Stress-Related DEGs

ROC analysis was used to evaluate the diagnostic values of gene expression levels in cancer tissues. The diagnostic values were better when the area under the curve (AUC) was closer to 1 [11, 15]. In LAC, the diagnostic values of oxidative stress-related DEGs (CCNA2, ERO1A, CDK1, PLK1, CDC25C, ITGB4, and GJB2) were investigated through the ROC analysis. Further, we constructed a nomogram of the oxidative stress-related DEGs with prognostic and diagnostic values.

### 2.7. Risk Score Model of the Oxidative Stress-Related DEGs

Univariate Cox regression analysis was performed to evaluate the relationship between the oxidative stress-related DEGs (*CCNA2*, *ERO1A*, *CDK1*, *PLK1*, *CDC25C*, *ITGB4*, and *GJB2*) and the prognosis of LAC patients. The screening standard was *P* < 0.05. Multivariate Cox regression analysis and AIC criteria were performed to screen the oxidative stress-related DEGs that independently influence the prognosis of patients with LAC. Subsequently, we constructed a risk score model [16, 17].

### 2.8. Verification of the Roles of the Risk Score Model and Construction of the Risk Model-Related Nomogram

Correlation analysis was performed to investigate the relationship between the expression levels of risk model genes (*ERO1A*, *CDC25C*, and *ITGB4*) and the risk score model. The expression levels of *ERO1A*, *CDC25C*, and *ITGB4*, and their relationship with the clinicopathological characteristics of patients with LAC in the high- and low-risk groups were explored and observed by scatter diagram and heat map. K-M survival and Cox regression analyses were performed to evaluate the relationship between the risk model and the OS of patients with LAC. The risk model-related nomogram was constructed based on multivariate COX regression analysis results.

### 2.9. Signaling Mechanisms Involved in the Risk Score Model

The GSEA (version: 4.1.0) software platform was used to analyze the BP, MF, CC, and signaling pathways of the DEGs. The gene expression data of 535 LAC patients in the TCGA database were grouped via the risk score and recorded as the high- and low-risk groups. The impact of the high- and low-risk groups on each gene set on the GSEA platform was explored to understand the signaling pathways involved in the risk score model. The running process was performed 1000-fold [18, 19]. Nominal (NOM) *P* was the screening standard for GSEA analysis.

### 2.10. Relationship between Risk Score Genes and Immune Cell Infiltration

ssGSEA analysis method was used to calculate the immune cell infiltration levels in the tissues with LAC. Spearman correlation analysis was used to explore the correlation between the expression levels of oxidative stress-related DEGs (*ERO1A*, *CDC25C*, and *ITGB4*) and the immune cell infiltration levels. Thereafter, the expression levels of LAC immune infiltrating cells in the high- and low-expression groups of *ERO1A*, *CDC25C*, and *ITGB4* were analyzed by the median expression values of *ERO1A*, *CDC25C*, and *ITGB4*.

### 2.11. Identification of Risk Score Model Gene Expression in LAC Tissues

In April 2022, we extracted the cancer tissues and adjacent normal tissues from 8 patients who underwent surgical treatment in our hospital and were diagnosed with LAC. All patients signed the informed consent. The study was reviewed and approved by the ethics committee of Taihe Hospital. The expression levels of *ERO1A*, *CDC25C*, and *ITGB4* in 8 LAC tissues and paired normal tissues were examined based on the standard PCR assays [19]. The primer sequences included as follows: *ERO1A* 5′-ATGACATCAGCCAGTGTGGA-3′ (forward); 5′-CATGCTTGGTCCACTGAAGA-3′ (reverse); *CDC25C* 5′-TGGTCACCTGGATTCTTC-3′ (forward); 5′-ACCATTCGGAGTGCTACA-3′ (reverse); and *ITGB4* 5′-TTCAATGTCGTCTCCTCCAC-3′ (forward); 5′-CAATAGGTCGGTTGTCATCG-3′ (reverse).

### 2.12. Statistical Analysis

The oxidative stress-related DEGs in LAC were analyzed by limma package or *t*-test. Survival and ROC analyses were performed to analyze the LAC prognosis and diagnostic value of the oxidative stress-related DEGs, as well as the roles of the risk model in the prognosis of LAC patients. Correlation analysis was conducted to explore the relationship between the expression of *ERO1A*, *CDC25C*, and *ITGB4* and LAC immune infiltration. *P* < 0.05 was considered statistically significant.

## 3. Results

### 3.1. Oxidative Stress-Related DEGs

A total of 32 gene sets related to oxidative stress were searched on the GSEA platform. These 32 gene sets comprised 784 OSRGs. The OSRGs in normal lung and LAC tissues were corrected and extracted from the TCGA database. Differential expression analysis showed 163 DEGs in LAC tissues compared to normal lung tissues (Table 1). Among them, 104 genes were overexpressed, whereas 59 were downregulated. The scatter plot displayed 8 overexpressed and 8 downregulated genes (Figure 1).

### 3.2. Functions, Mechanisms, and PPI Network of Oxidative Stress-Related the DEGs

GO annotation revealed that the oxidative stress-related DEGs contributed to the cellular response to oxidative stress, reactive oxygen species, toxic substance, antibiotics, hydrogen peroxide, metallic process, hydrogen peroxide, cellular oxidative detoxification, etc. (Figures 2(a)–2(c) and Table S1). KEGG analysis revealed that the oxidative stress-related DEGs are involved in the cell cycle, cellular sensitivity, endocrine resistance, *FOXO* signaling pathway, non-small-cell lung cancer, *TNF* signaling pathway, ferroptosis, transcriptional misregulation in cancer, *HIF-1*, *IL-17*, p53, and among other signaling pathways (Figure 2(d) and Table 2).  Figure 3(a) shows the PPI network between the oxidative stress-related DEGs and the enriched PPI networks through enrichment analysis (Figures 3(b)–3(d)).

### 3.3. Construction of the Prognostic Nomogram of Oxidative Stress-Related DEGs

K-M survival analysis showed that the expression levels of *BTK*, *CAT*, *CCNA2*, *CDC25C*, *CDH3*, *ERO1A*, *CDK1*, *PLK1*, *ITGB4*, *GJB2*, *CHEK1*, *CYBB*, *ECT2*, *FANCD2*, *FBLN5*, *GPR37*, *GPX3*, *GPX8*, *HMGA1*, *ITGAL*, *KCNA5*, *LRRK2*, *MCM4*, *MELK*, *MMP3*, *MMP14*, *MYBL2*, *NFIX*, *NOX4*, *NOX5*, *NUDT1*, *OAT*, *PRKAA2*, *PTPRN*, *RGS14*, *SELENBP1*, *SELENOP*, *SLC1A1*, *TRPA1*, *UBE2C*, and *XDH* significantly correlated with the poor prognosis of LAC patients (Table 3). Based on the significance criterion of the *P* < 0.001, the overexpression levels of *CCNA2*, *CDC25C*, *ERO1A*, *CDK1*, *PLK1*, *ITGB4*, and *GJB2* significantly correlated with the poor prognosis of patients with LAC (Figure 4).

ROC analysis demonstrated that the expression levels of *CCNA2*, *CDC25C*, *ERO1A*, *CDK1*, *PLK1*, *ITGB4*, and *GJB2* have diagnosis values of LAC (Figure 5). The AUCs of *CCNA2*, *CDC25C*, *ERO1A*, *CDK1*, *PLK1*, *ITGB4*, and *GJB2* were 0.97, 0.984, 0.984, 0.945, 0.984, 0.771, and 0.959, respectively, indicating that OSRGs *CCNA2*, *CDC25C*, *ERO1A*, *CDK1*, *PLK1*, *ITGB4*, and *GJB2* have diagnosis values of LAC. Based on K-M survival and ROC analyses, we constructed a nomogram of OSRGs *CCNA2*, *CDC25C*, *ERO1A*, *CDK1*, *PLK1*, *ITGB4*, and *GJB2* (Figure 6).

### 3.4. Construction of Risk Score Model

Univariate Cox regression analysis was used to explore the relationship between the expression levels of *CCNA2*, *CDC25C*, *ERO1A*, *CDK1*, *PLK1*, *ITGB4*, and *GJB2* and the OS of patients with LAC. Consequently, the overexpression of *CCNA2*, *CDC25C*, *ERO1A*, *CDK1*, *PLK1*, *ITGB4*, and *GJB2* was the risk factors for poor prognosis in patients with LAC (Figure 7(a)). Based on multivariate Cox regression analysis and the AIC method, *ERO1A*, *CDC25C*, and *ITGB4* were independent risk factors affecting the poor prognosis of patients with LAC (Table 4 and Figure 7(b)). The risk score model was constructed based on *ERO1A*, *CDC25C*, and *ITGB4*. Correlation analysis revealed that the expression levels of *ERO1A*, *CDC25C*, and *ITGB4* significantly correlated with the risk score (Figure S1A-C). Grouping by high- and low-risk showed significant differences between the two groups in *ERO1A*, *CDC25C*, and *ITGB4* (Figure S1D-F).

### 3.5. Risk Score as a Factor for Poor Prognosis in Patients with LAC

The expression levels of *ERO1A*, *CDC25C*, and *ITGB4* were significantly upregulated in LAC tissues from our hospital with significant statistical significance (Figure S2). Figures 7(c) and 7(d) show the relationship between risk score and OS of patients with LAC, and LAC with high-risk scores had a poor prognosis. Univariate Cox regression analysis showed that clinical stage, T stage, lymph node metastasis, and risk score affect the poor prognosis of patients with LAC (Figure 8(a)). Besides, multivariate Cox regression analysis revealed that age, clinical stage, and risk score contribute to the poor prognosis of patients with LAC (Figure 8(b)).  Figure 8(c) shows that the high- and low-risk groups are associated with the survival status, clinical stage, T stage, and lymph node metastasis in patients with LAC. To evaluate the prognosis of patients with LAC, a risk score prognostic nomogram was constructed based on multivariate Cox analysis results (Figure 9).

### 3.6. Signaling Mechanisms in a High-Risk Score Group

GSEA results showed that the high-risk score is involved in cell cycle, splice some, DNA replication, mismatch repair, homologous recombination, proteasome, nucleoside precision repair, p53 signaling pathway, base precision repair, oocyte meiosis, regulation of actin cytoskeleton, pathways in cancer, and among other mechanisms (Figure S3 and Table 5).

### 3.7. The Risk Score Model-Related DEGs Correlate with Immune Infiltrating Cells

Spearman correlation analysis demonstrated that the expression level of *CDC25C* correlated with the levels of Th2 cells, mast cells, iDC, eosinophils, DC, NK cells, Tfh, Tgd, NK cd56dim cells, CD8 T cells, macrophages, pDC, Tcm, Th17 cells, T helper cells, aDC, neutrophils, Tem, NK cd56bright cells, B cells, and Treg (Figure 10 and Table 6). *ERO1A* expression level correlated with Th2 cells, mast cells, eosinophils, Tfh, CD8 T cells, NK cd56dim cells, aDC, iDC, NK cells, NK cd56bright cells, Tgd, DC, pDC, neutrophils, and Treg (Figure S4 and Table 6). *ITGB4* expression level correlated with the NK cells, T helper cells, neutrophils, B cells, NK cd56bright cells, TFH, NK cd56dim cells, iDC, and mast cells (Figure S5 and Table 6).

Grouping by the median values of oxidative stress-related DEGs (*CDC25C*, *ERO1A*, and *ITGB4*) showed abnormal and statistically significant expression of mast cells, iDC, eosinophils, DC, NK cd56dim cells, NK cells, Tfh, Tgd, Th2 cells, macrophages, CD8 T cells, pDC, T helper cells, Th17 cells, Tcm, neutrophils, and Tem in the high- and low-expression groups of CDC25C (Figure 11 and Table 7). The expression of mast cells, iDC, eosinophils, CD8 T cells, NK cells, Tfh, Th2 cells, NK cd56bright cells, Tgd, aDC, T helper cells, NK cd56dim cells, DC, neutrophils, and B cells in the high- and low-expression groups of *ERO1A* was abnormal and statistically significant (Figure S6 and Table 7). The expression of NK cells, T helper cells, NK cd56bright cells, NK cd56dim cells, B cells, and neutrophils in the high- and low-expression groups of *ITGB4* was abnormal and statistically significant (Figure S7 and Table 7).

## 4. Discussion

Lung adenocarcinoma has a high incidence and mortality rates [7, 9, 15, 20]. At present, the prognosis of LAC patients is significantly poor. Therefore, new biomarkers are required to predict this and provide novel treatment targets. An oxidative stress response is involved in the progression of LAC [5–8]. Long-chain noncoding RNA (lncRNA) nuclear LUCAT1 (*NLUCAT1*) is strongly upregulated during hypoxia *in vitro* and is associated with hypoxia markers and poor prognosis in LAC. *NLUCAT1* downregulation inhibits the proliferation and invasion of LAC cells and increases oxidative stress and sensitivity to cisplatin [8]. Several OSRGs were abnormally expressed in LAC tissues in this study. The oxidative stress-related DEGs regulate the cellular response to oxidative stress, reactive oxygen species, toxic substances, antibiotics, hydrogen peroxide, reactive oxygen species, metabolic process, hydrogen peroxide, cellular oxidant detoxification, etc. This confirms that our oxidative stress-related DEGs are related to oxidative stress.

The expression levels of *CCNA2*, *CDC25C*, *ERO1A*, *CDK1*, *PLK1*, *ITGB4*, and *GJB2* could influence the cancer progression [21–26]. For instance, *ERO1A*, also known as *ERO1L,* promotes *IL6R* secretion by targeting disulfide bond formation. *IL-6R* binds to *IL-6*, resulting in the activation of the *NF-κB* signaling pathway. *NF-κB*, in turn, binds to the promoter of *MUC16*, causing its overexpression. *ERO1L* may trigger *CA125* secretion via the *IL-6* signaling pathway, form a positive feedback loop, and promote lung cancer development [23]. Through survival, ROC, and Cox analyses, we found that *CCNA2*, *CDC25C*, *ERO1A*, *CDK1*, *PLK1*, *ITGB4*, and *GJB2* significantly correlated with overexpression levels and poor prognosis of patients with LAC and exhibited diagnosis values of LAC. Bioinformatics analysis and PCR identification showed overexpressed oxidative stress-related DEGs *ERO1A*, *CDC25C*, and *ITGB4* in LAC tissues and were independent risk factors for poor prognosis in patients with LAC. The risk model based on *ERO1A*, *CDC25C*, and *ITGB4* is an independent risk factor for poor prognosis in patients with LAC. In the risk model-related nomogram, the risk score demonstrated the greatest impact on the prognosis of LAC patients. This indicates that our risk score model evaluates the prognosis of LAC patients.

Cell cycle, homologous recombination, and p53 signaling pathway are associated with cancer progression [27–31]. Cyclin B1 (*CCNB1*) is an important gene in mitosis and is upregulated in LAC tissues. *CCNB1* overexpression contributes to the advanced tumor stage and short OS. A negative correlation has been discovered between *miR-139-5p* and *CCNB1* expression levels. Through negative *CCNB1* regulation, *miR-139-5p* inhibits cell proliferation and migration [27]. lncRNA *CASC2* is downregulated in LAC. Its overexpression inhibits the proliferation of LAC cells and improves apoptosis. It also directly inhibits *miR-21* expression and upregulates p53 protein expression to mediate cell proliferation and apoptosis in LAC [31]. GSEA results showed that the high-risk score is implicated in cell cycle, DNA replication, homologous recombination, p53 signaling pathway, and other mechanisms in cancer progression. Our risk model based on the *ERO1A*, *CDC25C*, and *ITGB4* is closely related to the signaling mechanisms of cancer progression, preliminarily confirming that our risk model is closely associated with LAC progression.

In recent years, immunotherapy has been a crucial treatment option for patients with LAC [32–35]. Additionally, immunotherapy improves the clinical stage in patients with advanced cancer, hence providing them with an opportunity for surgery. Of note, the immune microenvironment is an important component in immunotherapy. For instance, *PD-1* and *PD-L1* blockers have been approved as standard therapy for non-small-cell lung cancer. In contrast with chemotherapy or radiotherapy, *PD-1*/*PD-L1* blocking therapy improves the remission rate. It prolongs the survival time, with fewer side effects in patients with advanced non-small-cell lung cancer treated with a single drug or combined therapy [32, 33]. NK cells act on targeted tumor cells, contributing to antitumor immunity. In non-small-cell lung cancer, there was an increase in the expression of immune checkpoint receptor *PD-1* on the surface of NK cells. In contrast with peripheral NK cells, the role of NK cells in tumor is poor, and this dysfunction is associated with the expression level of PD-1. PD-1 blocking therapy reverses the PD-L1-mediated inhibition of PD-1 NK cells [35]. We explored the relationship between the OSRGs *ERO1A*, *CDC25C*, and *ITGB4* expression levels and the immune microenvironment. As a result, the expression levels of *ERO1A*, *CDC25C*, and *ITGB4* significantly correlated with the levels of NK cells, mast cells, Tfh, NK cd56dim cells, iDC, neutrophils, and NK cd56bright cells. Nonetheless, additional future studies are necessary to confirm the roles of the OSRGs *ERO1A*, *CDC25C*, and *ITGB4* in the LAC immune microenvironment.

Our study applies bioinformatics analysis to investigate the roles of the OSRGs in the progression of LAC. The strengths of this study include large sample size, long follow-up time, and comprehensive prognostic data in the TCGA database. Besides, we provide novel candidate markers for LAC treatment and a risk model that evaluates the prognosis of LAC patients. Through PCR detection, *ERO1A*, *CDC25C*, and *ITGB4* expressions were significantly upregulated in the tissues from our hospital. Nevertheless, large amounts of tissues and patient prognostic data are necessary to verify the risk score model. Therefore, future studies should collect additional clinical tissue samples to detect the expression levels of *CDC25C*, *ERO1A*, and *ITGB4* and investigate their roles in the prognosis of LAC. Moreover, other research should explore the roles and mechanisms of *CDC25C*, *ERO1A*, and *ITGB4* in the immunity and progression of LAC at the cellular level.

## 5. Conclusion

In conclusion, *CCNA2*, *CDC25C*, *ERO1A*, *CDK1*, *PLK1*, *ITGB4*, and *GJB2* of OSRGs have diagnosis values of LAC and are associated with the prognosis of patients with LAC. *ERO1A*, *CDC25C*, and *ITGB4* overexpressions are independent risk factors for poor prognosis in patients with LAC. A high-risk score is an independent factor affecting the poor prognosis of LAC patients. *ERO1A*, *CDC25C*, and *ITGB4* expressions of risk score model genes significantly correlate with the levels of mast cells, IDC, NK cells, and CD8 T cells of LAC immune infiltrating cells. Therefore, the risk score model based on the *ERO1A*, *CDC25C*, and *ITGB4* is expected to predict the prognosis of patients with LAC.

## Figures and Tables

**Figure 1:** The DEGs associated with oxidative stress visualized with statistical significance: (a) overexpressed genes; (b) downregulated genes. Note: LAC: lung adenocarcinoma; DEGs: differentially expressed genes; ^∗∗∗^*P* < 0.001.

**Figure 2:** Functions and mechanisms of oxidative stress-related the DEGs using GO and KEGG analysis: (a) biological process; (b) cell composition; (c) molecular function; (d) signaling pathways. Note: DEGs: differentially expressed genes; BP: biological process; CC: cell composition; MF: molecular function; GO: Gene Ontology; KEGG: Kyoto Encyclopedia of Genes and Genomes.

**Figure 3:** PPI network of the oxidative stress-related DEGs. Note: PPI: protein-protein interaction; DEGs: differentially expressed genes.

**Figure 4:** 7 oxidative stress-related DEGs assess the overall survival of LAC: (a) *CDC25C*; (b) *GJB2*; (c) *ITGB4*; (d) *PLK1*; (e) *CCNA2*; (f) *ERO1A*; (g) *CDK1*. Note: LAC: lung adenocarcinoma; DEGs: differentially expressed genes.

**Figure 5:** 7 oxidative stress-related DEGs have diagnosis values of LAC: (a) *CDC25C*; (b) *GJB2*; (c) *ITGB4*; (d) *PLK1*; (e) *CCNA2*; (f) *ERO1A*; (g) *CDK1*. Note: LAC: lung adenocarcinoma; DEGs: differentially expressed genes.

**Figure 6:** Prognostic nomogram of 7 oxidative stress-related DEGs in LAC. LAC: lung adenocarcinoma; DEGs: differentially expressed genes.

**Figure 7:** Construction of risk model based on the 3 oxidative stress-related DEGs: (a) prognostic DEGs are shown in overall survival using COX analysis; (b) the relationship between 3 oxidative stress-related DEGs and prognosis in LAC; (c, d) the relationship between the risk score and prognosis in patients with LAC is visualized. Note: LAC: lung adenocarcinoma; DEGs: differentially expressed genes.

**Figure 8:** A risk score model based on the 3 oxidative stress-related DEGs is significantly associated with the prognosis in LAC patients. (a, b) COX analysis shows that risk score affects the poor prognosis of patients with LAC. (c) Risk score is associated with the survival status, clinical stage, T stage, and lymph node metastasis in patients with LAC. Note: LAC: lung adenocarcinoma; DEGs: differentially expressed genes.

**Figure 9:** Construction of the risk score prognostic nomogram.

**Figure 10:** The expression level of *CDC25C* correlates with the levels of immune infiltrating cells: (a) Th2 cells; (b) mast cells; (c) eosinophils; (d) NK cells; (e) iDC; (f) Tgd; (g) TFH; (h) DC; (i) NK CD56dim cells.

**Figure 11:** Abnormal expression of immune cells in the high- and low-expression groups of *CDC25C*: (a) Th2 cells; (b) Tgd; (c) eosinophils; (d) TFH; (e) NK CD56dim cells; (f) mast cells; (g) NK cells; (h) DC; (i) iDC.

**Table 1:** The oxidative stress-related DEGs in LAC tissues.

Gene	logFC	Gene	logFC	Gene	logFC	Gene	logFC
GPX2	6.013780623	SUMO4	2.257715062	PCNA	1.251080564	NFIX	-1.302326118
S100A7	5.41728031	FBXO32	2.253504422	PPIF	1.228327064	JUND	-1.316092598
MMP11	5.370660455	ERO1A	2.169220374	P4HB	1.224045072	SNCA	-1.343581323
GJB2	4.664130361	MMP9	2.153880308	CBX4	1.194091529	TLR4	-1.375114638
PTPRN	4.431031909	CDH2	2.13556165	GCLM	1.175006466	AQP1	-1.395667559
UBE2C	4.33254131	MT1H	2.048791978	UTP25	1.172874466	HMOX1	-1.474996851
WNT16	4.221055426	MARCKSL1	2.0461911	ERBB2	1.170033481	SESN1	-1.488992986
XDH	4.189103258	SLC4A11	2.023752334	SPINT2	1.147192812	ERBB4	-1.508245365
MMP3	4.042213517	PDK1	1.897233653	CALU	1.146319227	SELENOP	-1.513089809
MYBL2	3.97196672	ITGB4	1.769385266	RGS14	1.130235535	FOS	-1.547672977
CDC20	3.923133178	TXNRD1	1.713452233	NME2	1.120700065	KRT1	-1.611799687
PYCR1	3.849785485	FANCD2	1.694266871	GSR	1.118622392	BMP2	-1.62052111
CDC25C	3.822823814	WNT1	1.652280572	NUDT1	1.110791055	KLF2	-1.630982183
MELK	3.79228364	ABCB11	1.648035243	OAT	1.108313278	RCAN1	-1.645841006
CDKN2A	3.660292428	IGFBP2	1.643496508	TCF3	1.106493729	FBLN5	-1.650383453
PLK1	3.355128242	E2F1	1.629703342	IER3	1.104634685	ALOX5	-1.670847714
SLC7A11	3.206827355	GDF15	1.594567934	CDK4	1.1019358	MSRB3	-1.695874161
NOX5	3.181844416	FUT8	1.582037385	PARP1	1.097260888	EGR1	-1.730851757
NQO1	3.122327878	CYP2E1	1.575457932	MGST1	1.083753103	CHRNA4	-1.759665302
HGFAC	3.084341171	NOX1	1.572211162	NR2F6	1.077443474	CAT	-1.761079975
COL1A1	3.04475487	E2F3	1.541174573	DHFR	1.064060918	CYP1A1	-1.771485237
CCNA2	3.037368198	UCN	1.536180525	NOL3	1.017279978	HYAL1	-1.793702837
CDH3	2.906398001	PRDX4	1.524830048	HBB	-4.072278882	CRYAB	-1.799207942
GPR37	2.892829344	SRXN1	1.523512148	HBA2	-3.971614753	LRRK2	-1.837429368
SLC7A5	2.832579597	TPO	1.497068338	ETS1	-1.009611374	EDN1	-1.837496875
TRPA1	2.725732428	NET1	1.492518868	JUNB	-1.029141797	CA3	-1.923666594
EZH2	2.71140365	NOX4	1.469389165	ETV5	-1.03192463	SLC1A1	-2.043700892
SGK2	2.696077295	CBX8	1.467297358	ITGAL	-1.045741495	NR4A3	-2.088467157
CDK1	2.607317686	G6PD	1.459631279	VIM	-1.048813585	KCNA5	-2.103363458
CBX2	2.603102932	MET	1.424801169	CYGB	-1.072716336	GPX3	-2.12554072
LPO	2.537856476	FMO1	1.418278305	MYLK	-1.073347764	DUOX1	-2.428487405
E2F2	2.515712683	TRPM2	1.383090886	SIRPA	-1.104069804	HBEGF	-2.431447934
CDC25A	2.506554418	PRKAA2	1.373646285	SELENBP1	-1.12795438	EPAS1	-2.587591866
HMGA1	2.412891462	GPR37L1	1.36067259	CDKN2B	-1.146620037	IL6	-2.664089275
FOXO6	2.408776331	IPCEF1	1.347748923	CYBB	-1.155101406	CD36	-2.768036549
CHEK1	2.394961963	TAT	1.339357309	HYAL2	-1.155726104	AGRP	-2.793810482
GCLC	2.381107058	GPX8	1.337343767	NCF1	-1.157427085	RETN	-2.813480794
MCM4	2.359143052	MAP2K6	1.332194326	UTRN	-1.180127364	MGAT3	-2.885893674
ECT2	2.328988223	MMP14	1.302518357	BTK	-1.217464546	SCGB1A1	-3.072434982
EFNA4	2.310996951	TRAP1	1.281380934	PPARGC1B	-1.249251755	ANGPTL7	-3.157773456
HYOU1	1.280070739	BNIP3	1.270862371	HBA1	-4.201724914		

Note: LAC: lung adenocarcinoma; DEGs: differentially expressed genes.

**Table 2:** The mechanisms of the oxidative stress-related DEGs.

ID	Description	Adjust *P*	Count
hsa04110	Cell cycle	1.76724*E*-07	15
hsa04218	Cellular senescence	1.43121*E*-05	14
hsa05219	Bladder cancer	1.43121*E*-05	8
hsa05144	Malaria	5.35207*E*-05	8
hsa05166	Human T-cell leukemia virus 1 infection	6.57929*E*-05	15
hsa05418	Fluid shear stress and atherosclerosis	6.57929*E*-05	12
hsa00480	Glutathione metabolism	8.24298*E*-05	8
hsa01522	Endocrine resistance	8.24298*E*-05	10
hsa05225	Hepatocellular carcinoma	0.000314944	12
hsa04068	FoxO signaling pathway	0.000873542	10
hsa05223	Non-small-cell lung cancer	0.002645764	7
hsa04933	AGE-RAGE signaling pathway in diabetic complications	0.003188844	8
hsa05161	Hepatitis B	0.00397965	10
hsa04668	TNF signaling pathway	0.005960585	8
hsa04216	Ferroptosis	0.006375126	5
hsa05215	Prostate cancer	0.010743162	7
hsa05202	Transcriptional misregulation in cancer	0.010743162	10
hsa04380	Osteoclast differentiation	0.010743162	8
hsa05218	Melanoma	0.010743162	6
hsa04918	Thyroid hormone synthesis	0.012331107	6
hsa05206	MicroRNAs in cancer	0.012331107	13
hsa05212	Pancreatic cancer	0.012331107	6
hsa05169	Epstein-Barr virus infection	0.012694013	10
hsa04066	HIF-1 signaling pathway	0.015124736	7
hsa05224	Breast cancer	0.019724031	8
hsa05226	Gastric cancer	0.02063717	8
hsa05143	African trypanosomiasis	0.021418019	4
hsa00590	Arachidonic acid metabolism	0.023628458	5
hsa04934	Cushing syndrome	0.023628458	8
hsa05022	Pathways of neurodegeneration-multiple diseases	0.023993575	16
hsa04657	IL-17 signaling pathway	0.025867689	6
hsa05230	Central carbon metabolism in cancer	0.033496361	5
hsa05205	Proteoglycans in cancer	0.034153721	9
hsa04115	p53 signaling pathway	0.037682051	5
hsa05214	Glioma	0.041022366	5
hsa05220	Chronic myeloid leukemia	0.042160826	5
hsa05140	Leishmaniasis	0.043324911	5
hsa05167	Kaposi sarcoma-associated herpesvirus infection	0.065724291	8
hsa00130	Ubiquinone and other terpenoid-quinone biosynthesis	0.069783669	2
hsa05222	Small-cell lung cancer	0.082734228	5
hsa05323	Rheumatoid arthritis	0.084248714	5

Note: DEGs: differentially expressed genes.

**Table 3:** The expression levels of oxidative stress-related DEGs are significantly correlated with the poor prognosis of LAC patients.

Gene	*P*	Gene	*P*	Gene	*P*
BTK	1.493*e*-03	GPX3	1.072*e*-02	NOX5	2.935*e*-02
CAT	1.529*e*-02	GPX8	5.265*e*-03	NUDT1	2.177*e*-02
CCNA2	9.186*e*-05	HMGA1	3.920*e*-03	OAT	3.028*e*-02
CDC25C	3.027*e*-04	ITGAL	2.305*e*-02	PLK1	3.684*e*-04
CDH3	4.037*e*-02	ITGB4	8.341*e*-04	PRKAA2	4.034*e*-02
CDK1	1.854*e*-04	KCNA5	8.226*e*-03	PTPRN	3.107*e*-02
CHEK1	3.871*e*-03	LRRK2	4.389*e*-02	RGS14	6.938*e*-03
CYBB	3.658*e*-02	MCM4	6.422*e*-03	SELENBP1	2.610*e*-02
ECT2	4.329*e*-03	MELK	3.742*e*-02	SELENOP	2.561*e*-02
ERO1A	3.599*e*-04	MMP3	1.822*e*-02	SLC1A1	3.487*e*-02
FANCD2	2.336*e*-02	MMP14	3.558*e*-02	TPRA1	4.763*e*-03
FBLN5	4.130*e*-02	MYBL2	3.134*e*-02	UBE2C	4.573*e*-02
GJB2	1.853*e*-04	NFIX	1.384*e*-02	XDH	4.819*e*-02
GPR37	9.159*e*-03	NOX4	1.578*e*-02		

Note: LAC: lung adenocarcinoma; DEGs: differentially expressed genes.

**Table 4:** Independent prognostic factors of oxidative stress-related DEGs.

Gene	HR	95% CI	*P*
ERO1A	1.363360001	1.124731516-1.652617062	0.001592209
CDC25C	1.459214408	1.138311378-1.870583683	0.002860696
ITGB4	1.16932949	1.039123642-1.315850589	0.009400705

Note: DEGs: differentially expressed genes; HR: hazard ratio; CI: confidence interval.

**Table 5:** Signaling mechanisms are involved in the high-risk score group.

Name	Size	ES	NES	NOM *P*
Cell cycle	124	0.66915077	2.1871314	0
Spliceosome	126	0.64206976	2.083224	0
DNA replication	36	0.837718	2.0672143	0
Mismatch repair	23	0.80036765	2.062228	0
Pathogenic Escherichia coli infection	55	0.5739781	2.056669	0
Homologous recombination	28	0.7681676	2.0361679	0
P53 signaling pathway	68	0.49579692	1.8950231	0
Pyrimidine metabolism	97	0.5173413	1.9280515	0.001923077
Nucleotide excision repair	44	0.6324002	1.995188	0.001980198
Base excision repair	33	0.6285262	1.8693517	0.002
Proteasome	44	0.7988379	2.0141854	0.002040816
Oocyte meiosis	112	0.4684853	1.8251096	0.004140787
Pentose phosphate pathway	27	0.57422036	1.7523918	0.005825243
Glycolysis gluconeogenesis	61	0.50060135	1.7604159	0.01010101
Ubiquitin mediated proteolysis	133	0.4287824	1.6589828	0.018907564
Bladder cancer	42	0.39720345	1.5345889	0.02296451
Pancreatic cancer	70	0.41440853	1.598584	0.024948025
Small-cell lung cancer	84	0.41004965	1.5795516	0.02631579
Galactose metabolism	25	0.50981605	1.6308589	0.027985075
Renal cell carcinoma	70	0.37961188	1.518121	0.028077753
Regulation of actin cytoskeleton	212	0.37622863	1.5810093	0.028688524
Drug metabolism other enzymes	51	0.4489914	1.5682174	0.029850746
Pathways in cancer	325	0.31233284	1.4214869	0.042105265
Progesterone mediated oocyte maturation	85	0.3916816	1.5144613	0.04375

Note: ES: enrichment score; NES: normalized enrichment score; NOM: nominal.

**Table 6:** The expression levels of oxidative stress-related DEGs are correlated with the levels of immune infiltrating cells in LAC.

Immune cells	CDC25C (*r*)	*P*	ERO1A (*r*)	*P*	ITGB4 (*r*)	*P*
aDC	0.121	0.005	0.174	<0.001	0.061	0.159
B cells	-0.095	0.027	-0.081	0.061	-0.156	<0.001
CD8 T cells	-0.195	<0.001	-0.210	<0.001	0.078	0.070
Cytotoxic cells	-0.008	0.847	-0.015	0.737	-0.054	0.217
DC	-0.277	<0.001	-0.130	0.003	0.074	0.088
Eosinophils	-0.347	<0.001	-0.236	<0.001	0.071	0.102
iDC	-0.352	<0.001	-0.164	<0.001	0.091	0.035
Macrophages	-0.173	<0.001	0.034	0.431	0.049	0.257
Mast cells	-0.517	<0.001	-0.354	<0.001	0.087	0.044
Neutrophils	-0.115	0.008	0.096	0.027	0.162	<0.001
NK CD56bright cells	-0.101	0.019	-0.139	0.001	0.128	0.003
NK CD56dim cells	0.211	<0.001	0.178	<0.001	0.097	0.026
NK cells	-0.238	<0.001	-0.163	<0.001	0.255	<0.001
pDC	-0.152	<0.001	-0.110	0.011	0.010	0.823
T cells	-0.070	0.105	-0.022	0.610	-0.085	0.050
T helper cells	0.135	0.002	0.084	0.053	-0.196	<0.001
Tcm	-0.151	<0.001	-0.049	0.258	-0.020	0.638
Tem	-0.107	0.013	-0.007	0.870	-0.025	0.566
TFH	-0.236	<0.001	-0.222	<0.001	-0.104	0.017
Tgd	0.220	<0.001	0.137	0.001	-0.051	0.235
Th1 cells	-0.040	0.353	0.076	0.077	-0.002	0.954
Th17 cells	-0.143	<0.001	-0.063	0.144	0.080	0.066
Th2 cells	0.771	<0.001	0.464	<0.001	-0.073	0.092
TReg	0.091	0.036	0.091	0.036	0.082	0.057

Note: LAC: lung adenocarcinoma; DEGs: differentially expressed genes.

**Table 7:** The levels of immune infiltrating cells are differentially expressed in the groups of oxidative stress-related DEGs.

Immune cells	CDC25C (*P*)	ERO1A (*P*)	ITGB4 (*P*)
aDC	0.065	0.003	0.35
B cells	0.069	0.038	0.009
CD8 T cells	0.001	0	0.089
Cytotoxic cells	0.961	0.871	0.372
DC	0	0.008	0.678
Eosinophils	0	0	0.815
iDC	0	0	0.254
Macrophages	0.001	0.719	0.681
Mast cells	0	0	0.549
Neutrophils	0.04	0.02	0.047
NK CD56bright cells	0.139	0.001	0.001
NK CD56dim cells	0	0.007	0.003
NK cells	0	0	0
pDC	0.001	0.079	0.801
T cells	0.296	0.732	0.112
T helper cells	0.006	0.005	0
Tcm	0.028	0.893	0.299
Tem	0.044	0.902	0.959
TFH	0	0	0.205
Tgd	0	0.002	0.449
Th1 cells	0.452	0.052	0.974
Th17 cells	0.009	0.503	0.052
Th2 cells	0	0	0.926
TReg	0.051	0.269	0.065

Note: DEGs: differentially expressed genes.

## Data Availability

Our data can be obtained from the website of the TCGA database or by contacting the corresponding author.

## Abbreviations

OSRGs: Oxidative stress-related genes
LAC: Lung adenocarcinoma
GSEA: Gene Set Enrichment Analysis
DEG: Differentially expressed genes
IL-8: Interleukin-8
ROS: Reactive oxygen species
BC: Breast cancer
EMT: Epithelial-mesenchymal transformation
*Nrf2*: Nuclear factor, erythroid-derived 2
TCGA: The Cancer Genome Atlas
ROC: Operating characteristic
FDR: False discovery rate
OS: Overall survival.

## Supplementary Materials

Supplementary Materials Figure S1: the expression levels of oxidative stress-related the DEGs significantly correlate with the risk score. Note: LAC: lung adenocarcinoma; DEGs: differentially expressed genes. Figure S2: identification of risk model gene expression in LAC tissues. (A) ERO1A; (B) CDC25C; (C) ITGB4. Note: LAC: lung adenocarcinoma. Figure S3: the mechanisms of oxidative stress related to the DEGs. Note: DEGs: differentially expressed genes. Figure S4: the expression level of *ERO1A* correlates with the levels of immune infiltrating cells. Figure S5: the expression level of *ITGB4* correlates with the levels of immune infiltrating cells. Figure S6: abnormal expression of immune cells in the high- and low-expression groups of *ERO1A*. Figure S7: abnormal expression of immune cells in the high- and low-expression groups of *ITGB4*. Table S1: functions of oxidative stress-related the DEGs. Note: BP: biological process; CC: cell composition; MF: molecular function.
